The article "Data Visualization and Interaction of Urban Traffic Logistics Management System Using WebGIS" was published in 2022. Journal: Comput Intell Neurosci.

# Data Visualization and Interaction of Urban Traffic Logistics Management System Using WebGIS

**DOI:** 10.1155/2022/9347247

**Published:** 2022-06-27

**Authors:** Zhaodi Li, Dan Li

**Affiliations:** Industrial Design Engineering, Kunming University of Science and Technology, Kunming 650000, China

## Abstract

At present, the large amount of data generated by transportation and logistics in cities brings great difficulties to data management and operation. The purpose is to explore the applicability of WebGIS and expand the application of intelligent interactive urban traffic logistics management. An urban traffic logistics management system is designed for urban traffic route assignment and intelligent interaction based on the WebGIS system and the basic principles and related algorithms of urban traffic route assignment. Then, the operation of the system under different shortest path algorithms and different path assignment algorithms is discussed. As a result, the Dijkstra algorithm runs faster than the Floyd algorithm. The comparison of three different road assignment algorithms shows that the no road assignment algorithm has the smallest average time consumption, which is 264.43 ms. The running time of the continuous average algorithm is the same as that of the user balance algorithm. The WebGIS system has practical application value compared with the TransCAD system and Cube system. This article proposes that the interactive function of the system can be used normally. The vehicle information of the test sample points can be displayed, and the function realization effect is good. The research results can provide scientific references for the follow-up research on intelligent transportation.

## 1. Introduction

The development of transportation depends on the level of national and regional economic development. Traffic connectivity has become an important link within the national regional economic circle [1]. Moreover, with the acceleration of urbanization, the number of urban vehicles has increased year by year, and the existing traffic management system in China has been under great transport pressure [2]. Transportation planning is an important means to fully utilize limited transportation infrastructure, scientifically manage urban traffic, and solve traffic congestion [3]. Traffic planning is based on traffic demand forecasting technology to predict the relationship between future cities and traffic development, guiding the layout and construction of urban traffic network planning. The traditional traffic demand forecasting is complex and is subject to many restrictions [4]. Traffic demand forecasting software can be developed based on GIS (Geographic Information System) with the rapid development of CT (computer technology), IoT (Internet of Things), and AI (artificial intelligence) technologies, such as ML (Machine Learning), and intelligent traffic forecasting and management have become the focus of academic attention [5].

WebGIS technology has become the concern of researchers. WebGIS technology is the method of running GIS technology in the web (World Wide Web). It can use GIS analysis technology through the Internet without the local installation of GIS software [6]. Driven by the rapid development of the Internet, WebGIS is widely used and has become one of the critical technologies in social development [7]. WebGIS is being integrated with IT (information technologies), such as parallel computing, cloud computing, MI (Mobile Internet), IoT, UAVs (unmanned aerial vehicles), voice interface, ML, and AI, and is being applied in cutting-edge fields, including big data, smart cities, smart communities, smart commerce, unmanned driving, VR (virtual reality), and AR (augmented reality). WebGIS plays an important role in traffic management, and intelligent traffic forecasting, management, and interaction are essential in traffic management. Information interaction system is an important component of an ITS (intelligent transportation system). Most vehicle-road coordination functions in ITS are based on information interaction. More and more traffic information will be collected and integrated with the rapid development of wireless communication technology. Based on the collected information, the ITS of pedestrians, vehicles, and roads can be established to improve the efficiency, safety, and sustainability of the transportation system. This is of great significance for the realization of intelligent transportation. Makino et al. used intelligent transportation systems to study urban traffic problems. The research results revealed that the intelligent transportation system used information and communication technology to solve road traffic problems and could effectively solve various urban traffic problems [8]. Göhlich et al. comprehensively evaluated the transportation system based on system cost, energy demand, and transit time. It was found that the overall cost of the system could be reduced by 13% to 18% [9]. Zhao et al. used a WebGIS system for near-real-time disaster assessment and emergency response research, indicating that the proposed framework was powerful and proficient in automatically generating seismic deformation maps within minutes of an earthquake [10]. In conclusion, current research on ITS requires a data-driven approach to modeling. This article studies the construction of the traffic intelligent interactive system based on WebGIS technology. The value is that it can improve the digital degree of the urban traffic system.

The purpose of this article is to research the optimization and data visualization of the urban intelligent transportation logistics management system based on WebGIS technology. Research is based on existing Internet, artificial intelligence technologies, and traffic management systems. A new traffic logistics management system is designed using WebGIS. The system is optimized from the system architecture and shortest path design. The traffic logistics management system is constructed through the traffic distribution algorithm, the design algorithm of the shortest path in traffic. The innovation is to use WebGIS and B/S architecture to build the system. The main contribution is to propose a vehicle data transmission module to construct a traffic monitoring network. Through the comparison, the implementation effect of the designed system is fully explored, which has important reference value for the digital and intelligent development of the urban transportation system.

## 2. Principle and Method of Road Traffic System

### 2.1. Architecture of WebGIS

In the process of model building of road traffic systems, the architecture based on WebGIS can provide technical support and guarantee. GIS is a geographic software that is widely used in many fields, including urban planning, public transportation, and satellite remote sensing. However, with the continuous growth of information data, the traditional GIS has become incapable, showing high development costs, low maintenance efficiency, and high hardware requirements [11]. Hence, WebGIS appears. WebGIS is a combination of GIS and Internet technology, and it is also an extension of GIS, sharing spatial data on the web through the Internet. It can not only analyze and manage spatial data through GIS technology but also publish information and share data through Internet technology. It can not only analyze and manage spatial data through GIS technology but also publish information and share data through Internet technology [12]. Users can further develop functions, such as maps, geographic retrieval, and corresponding spatial analysis, which have practical value [13].

WebGIS architecture consists of terminal GIS mode, C/S (client/server) mode, and B/S (browser/server) mode. Here, the most widely used B/S mode is selected as the WebGIS architecture [14]. This mode has strong distribution and simple and convenient business expansion and can easily complete the synchronization update of users, as shown in Figure 1.

Figure 1 shows that the B/S structure is divided into three layers, namely, the client, the intermediate layer, and the data layer. The client can be developed through various WebGIS APIs (Application Programming Interface) to interact with GIS servers or business logic servers and provide users with web applications [15]. The intermediate layer includes the GIS servers and business logic servers. GIS servers can be open-source GIS projects, professional GIS development platforms, and Internet application map servers [16]. The intermediate layer can provide map data service and functional services for the application layer. The data layer provides basic data support, such as spatial data and business data. In B/S architecture, users do not have to configure multitier application software on the client-side, thus avoiding the complex and long structure in C/S architecture. Besides, users manage and maintain the database [17]. Servers can provide services through procedure call on the corresponding program to process data no matter data are accessed through what platform. Overall, the B/S architecture is more convenient to maintain and upgrade, has more diverse user groups, and has easier system access, popularizing the WebGIS.

### 2.2. WebGIS Development Plan

System development requires the selection of many WebGIS projects. Here, development libraries, servers, and databases are selected and researched from WebGIS clients. The current mainstream development libraries include OpenLayers and OpenScales. OpenScales is a front-end map framework based on ActionScript3 and Flex, supporting standard map services. Besides, it is often used to develop various web, mobile, and desktop map programs. It is also an open-source and free client-side development architecture and is used in various browsers, showing good cross-platform features. Therefore, the OpenScales architecture is chosen here [18]. The widely used GeoServer is selected for the WebGIS server. The users can update, delete, modify, and query the spatial database online through GeoServer. The server also supports multiple formats of data and projections. GeoServer is also free and open-source code, which is very efficient. The chosen spatial database is PostGIS, which supports several spatial data types such as point, line, polygon, multipoint, and multiline. It supports all data access and construction methods and includes features, such as spatial analysis, data support, and coordinate transformation.

### 2.3. Theoretical Basis of Dijkstra Shortest Path Algorithm

The shortest path refers to the path with the smallest sum of side weights between two points. The shortest path algorithm is an important theoretical basis for urban traffic management [19]. At present, popular shortest path algorithms include the Dijkstra algorithm, Bellman–Ford algorithm, Floyd algorithm, and SPFA algorithm. Here, the Dijkstra algorithm is selected [20].

The Dijkstra algorithm calculates the minimum impedance between two points or the minimum impedance between a node and any node. The calculation steps are shown below.

All the node features in the road traffic network are counted, and the marking equations are as follows:

(1) $$\begin{array}{c} P\left(a\right)=0, \end{array}$$

(2) $$\begin{array}{c} T_{1}\left(j\right)=\infty ,j=1,2,\ldots ,n, \end{array}$$

(3) $$\begin{array}{c} T_{k}\left(j\right)=m. \end{array}$$

In (1)–(3), *a* represents the starting point. *P* represents the starting point number. The other points are numbered as *T*. *n* represents the total number of sample nodes. *m* represents the weight coefficient of each node.

Then, suppose that after *K* − 1 step, the *i*th node is a point labeled with *P*. Then, in the *K*-step search, all the point *i* without a label is found and updated with label *T*, and the following equation can be obtained:

(4) $$\begin{array}{c} T_{k}\left(j\right)=\text{min}\left[T\left(j\right),P\left(i\right)+d_{ij}\right], \end{array}$$

where *d*_*ij*_ represents the weight from *i* to *j* and *T(j)* denotes the label *T* of point *j* before being marked.

After the *T* label is updated, the minimum value will be obtained in all *T* labels, and the following equation will be obtained:

(5) $$\begin{array}{c} T_{k}\left(j_{0}\right)=\min\left[T_{k}\left(j\right),T\left(r\right)\right], \end{array}$$

where *j*_0_ denotes the node number corresponding to the minimum *T* label and *T(r)* represents the label *T* of node *r* not adjacent to point *i*.

Afterward, the node with the minimum *T* labels will be updated with the *P* label, and the following equation will be obtained:

(6) $$\begin{array}{c} P\left(j_{0}\right)=T_{k}\left(j_{0}\right). \end{array}$$

When the *T* labels of all nodes become *P* labels, the Dijkstra algorithm ends.

In practice, the traffic volume in the traffic network is connected to the road network through the virtual road, namely, the centroid connecting rod; the centroid connecting rod needs to be calculated for correct results. Centroid is the node of the road traffic network. Centroid connecting rod is the line segment connecting centroid and general road network. Centroid and centroid connecting rods can concentrate the travel and attraction of the traffic area on a point and then quickly disperse the traffic volume to the traffic network, reducing the complexity of traffic allocation and workload [21, 22], as shown in Figure 2.

In Figure 2, the red dot is the centroid, while the gray imaginary line is the centroid connecting rod, and the black line is the formed road network. Here, the dynamic impedance calculation method can calculate the shortest path of the centroid connecting rod. The shortest path of connecting rod with centroid has the following characteristics: firstly, the time of vehicle passing through the centroid connecting rod is usually much less than that of ordinary road. Secondly, the shortest path in the traffic cell has and can only have two centroid connecting rods. Hence, the impedance of the centroid connecting rod should be a function of the flow, and a maximum function should be added at the end of the function. The specific content is as follows:

(7) $$\begin{array}{c} T_{Z}\left(v\right)=f\left(v\right)+C, \end{array}$$

where *T*_*z*_*(v)* is the resistance of the centroid link, *f(v)* represents the function of time and flow, and *C* denotes the maximum value, which is either a constant or a variable; the value is greater than the maximum impedance value in the general road section.

### 2.4. Theories of the Traffic Allocation Algorithm

The traffic assignment algorithm is a very important factor to be considered. Here, the analysis focus is on the all-and-nothing algorithm, the continuous average algorithm, and the user balance algorithm.

The all-and-nothing algorithm is the most basic traffic assignment algorithm. The algorithm assumes that the vehicle is not affected by traffic load, and road network congestion factors are not considered. The constant is used as the road resistance function [23]. This algorithm is simple in the calculation but results in uneven traffic volume distribution. All traffic volumes are concentrated on the shortest path, limiting its usage scope. The calculation steps are as follows. Firstly, the flow of all sections of the road network is set to 0, and the impedance of free driving is obtained. Secondly, the shortest path is obtained through the shortest path algorithm. Finally, matrix *T* is loaded into the corresponding road section according to the shortest path [24].

The continuous average algorithm continuously adjusts the flow of each road section through the weighted average to gradually approximate equilibrium [25]. The calculation steps are as follows.

The iteration number is set to 0, and the expression of the road resistance function can be expressed as follows:

(8) $$\begin{array}{c} C_{a}^{0}=C_{a}\left(0\right). \end{array}$$

The initial solution is obtained through the all-and-nothing allocation of the impedance during free driving.

Here is the research hypothesis:

(9) $$\begin{array}{c} n=n+1. \end{array}$$

Roadblocks are updated according to current traffic assignments:

(10) $$\begin{array}{c} C_{a}^{0}=C_{a}\left(x_{a}^{n-1}\right). \end{array}$$

The weighted average method can calculate the allocated current traffic volume *F*_*a*_^*n*^, as shown in the following equation:

(11) $$\begin{array}{c} x_{a}^{n}=\left(1-a\right)x_{a}^{n-1}+F_{a}^{n}. \end{array}$$

If there is little difference between *x*_*a*_^*n*−1^ and *x*_*a*_^*n*^, that is, if the following equation holds:

(12) $$\begin{array}{c} \frac{\sqrt{\sum_{a}x_{a}^{n+1}-x_{a}^{n}}}{\sum_{a}x_{a}^{n}}<\varepsilon , \end{array}$$

then the calculation is over, and otherwise, the roadblock will be updated.

In the user balance algorithm, all selected paths have the same impedance, and the impedances of unselected paths are greater than or equal to the selected path impedance [26]. It is calculated through the Beckmann model, as shown in the following equation [27]:

(13) $$\begin{array}{c} \min z\left(x\right)=\sum_{a}\int_{0}^{x_{a}}t_{a}\left(w\right)\text{d}w,\\ \text{s.t}\left\{\begin{array}{c} \sum_{k}f_{k}^{rs}=q_{rs},\\ f_{k}^{rs}\geq 0. \end{array}\right. \end{array}$$

Suppose that the constraint of the Beckmann model must be linear, and the solution of the model can be obtained through the FW algorithm. The specific steps are as follows. The first is to initialize the algorithm, as shown in the following equation:

(14) $$\begin{array}{c} t_{a}^{n}=t_{a}\left(0\right),\;\forall a. \end{array}$$

Traffic at each segment is expressed as in the following equation:

(15) $$\begin{array}{c} \left[x_{a}^{1}\right],\;\forall a. \end{array}$$

Then, the load impedance is updated according to traffic distribution, and the following equation can be obtained:

(16) $$\begin{array}{c} t_{a}^{n}=t_{a}\left(x_{a}^{n}\right),\;\forall a. \end{array}$$

Nearby traffic volume is obtained according to updated impedance. Then, the optimal iterative step length is determined, as expressed in the following equation:

(17) $$\begin{array}{c} \sum_{a}\left(y_{a}^{n}-x_{a}^{n}\right)t_{a}\left[x_{a}^{n}+\left(y_{a}^{n}-x_{a}^{n}\right)\right]=0. \end{array}$$

The new starting point of iteration is expressed as

(18) $$\begin{array}{c} x_{a}^{n+1}=x_{a}^{n}+\lambda \left(y_{a}^{n}-x_{a}^{n}\right). \end{array}$$

Finally, the convergence is tested, and if the following equation holds:

(19) $$\begin{array}{c} \frac{\sqrt{\sum_{a}{\left(x_{a}^{n+1}-x_{a}^{n}\right)}^{2}}}{\sum_{a}x_{a}^{n}}<\varepsilon , \end{array}$$

then it is proved that the new starting point of iteration meets the requirements, and the algorithm will stop. On the contrary, the update operation of road impedance is repeated.

### 2.5. Realization of Urban Transportation Logistics Management System

Thus, the urban traffic logistics management system is designed based on the above theories and architecture. The main functional modules of the system are divided as shown in Figure 3.

The system contains web basic functional modules and WebGIS traffic logistics management modules. The web basic module is the foundation of logistics management program and can provide users with system introduction, registration, and login operation. The web GIS traffic logistics management module is the core of the system, containing six submodules: basic information input, shortest path query, data file upload, shortest path calculation allocation, visualization, and information output. The users can call the map online, use the functions of the road network map, upload the normal function files, query the shortest path, and realize the intelligent interaction of the system.

The database can store user information and operating data. The MySQL database is selected as the relational database in the designed system [28]. MySQL database can store personal information, such as user name and password. Research shows that the MySQL database has limited spatial analysis capacity, so the PostgreSQL database is selected as the structural database of the system [29].

Here, road network information is analyzed, and data visualization is optimized. At the same time, a simple and beautiful user interface should be designed [30]. The visualization function module is divided into two parts, namely, road parameter setting and traffic saturation setting. The road parameter settings include the color, transparency, and width settings of the road. The users can set the pop-up color setting panel to visually select the required color [31]. Traffic saturation is the ratio of traffic volume to capacity. The default values of 0.3, 0.7, 0.8, and 0.9 are set as nodes and correspond to 1–5 grade line styles, respectively.

### 2.6. Interactive System Design

To optimize the application of the system, the system visualization function is expanded into a data aggregation platform for vehicle information through the IoT, wireless transmission technology, WebGIS technology, and web technology [32]. The overall architecture of the interactive system consists of field monitoring terminals, monitoring center networking, and remote application client, as shown in Figure 4.

The monitoring terminal is composed of ETC (electric toll collection)-II, IoT experimental platform, and data transmission module. It can read vehicle information in real-time and pack and transmits data to the monitoring center network [33]. The functions of the WebGIS interactive system are manifested through networking. After the real-time data packets of the on-site monitoring terminal are received, a series of works will be completed through networking, including data parsing, management, analysis, processing, storage, and visualization. Servers are configured through monitoring center networking. The remote application client can provide a PC client, mobile terminal, and smartphone with different functions according to the permission level [34].

The main functional modules of the interactive system are shown in Figure 5.

Figure 5 illustrates that the system contains three main functional modules, which are the system management module, data management module, and vehicle information display module. The interactive system is managed by administrators through the system management module, and the administrators can operate, maintain, and update the system, or add and delete system functions, set user permissions, and manage users. The collected data are managed by the data management module through operations, such as data processing, data backup, data import, data cleaning, data recovery, and data download. The vehicle information display module is the main functional module of the system, which is also the main function of the interactive system. The users can query the site location information and the real-time vehicle sample data of the simulated sites or view, zoom in, zoom out, drag, and drop the network map.

### 2.7. Experimental Parameter Settings

A simple road traffic system with two paths is designed to verify the road assignment function of different traffic assignment algorithms. The basic parameter data of the road network are obtained from the Mattzou database. The basic parameters of the two paths are listed in Table 1.

## 3. System Function Test Results

### 3.1. Function Realization under Different Traffic Allocation Algorithms

Here, three road traffic allocation methods are analyzed, namely, all-and-nothing, continuous average, and user balance methods. The changes of flow and impedance between road networks under three modes are measured, as shown in Figures 6 and 7.

Figures 6 and 7 demonstrate that in the all-and-nothing allocation algorithm, all traffic is loaded into a path 1#, which is consistent with the total travel volume of the road. Under this algorithm, the initial total impedance of 1# path and 2# path is 11.87 and 11.33, respectively. Hence, the allocation function of the all-and-nothing algorithm runs normally and meets expectations. Under the continuous average algorithm, the flow allocated on the 1# path and the 2# path is 66 and 136, respectively, and the sum of the two is 20 and is greater than the initial value. After allocation, the total impedance of 1# path and 2# path is 11.89 and 11.35, respectively, which is not balanced. Under the user allocation algorithm, the traffic on the 1# path and the 2# path are 119 and 81, respectively, and the sum of the two is 200. At the same time, the total impedance values on the two paths are 11.60, reaching the equilibrium condition.

### 3.2. Running Time of Shortest Path Algorithm

Based on the above allocation results, the running speed of the Dijkstra shortest path algorithm under different allocation algorithms is calculated. To verify the application effect of the Dijkstra shortest path algorithm, the running time of the Floyd algorithm is also analyzed and compared. The specific results of the all-and-nothing algorithm, continuous average, and user balance algorithm are shown in Figures 8(a)–8(c).

The average running times of eight experiments and different allocation algorithms are obtained, as shown in Figure 9.

Figure 9 implies that the running times of the Dijkstra shortest path algorithm among the three path assignment algorithms are 242.46 ms, 279.85 ms, and 266.86 ms, respectively. The running times of the Floyd shortest path algorithm among the three path assignment algorithms are 286.39 ms, 424.83 ms, and 426.92 ms, respectively. Therefore, the Dijkstra algorithm has a short running time and runs fast, which has significant advantages. The comparison of three different path assignment algorithms shows that the all-nothing algorithm has an average total time of 264.43 ms and the shortest running time. The running times of the continuous average algorithm and the user balance algorithm are 352.34 ms and 346.89 ms, respectively, and the two algorithms run at almost the same speed. The performance of the Dijkstra algorithm proposed here is the best in terms of road assignment time and system running speed. The innovation of the algorithm is to improve the running speed of the original algorithm.

### 3.3. Advantages of Traffic Allocation System Based on webGIS

The Dijkstra algorithm is used as the shortest path calculation to further verify the applicability of the traffic assignment system based on WebGIS. The popular TransCAD system and Cube are compared to explore the traffic allocation results under the all-and-nothing path assignment algorithm, continuous average algorithm, and user balance algorithm.

The results under the full all-and-nothing path allocation algorithm are shown in Figure 10.

Figure 10 shows that the allocation results of each system are completely consistent under the all-and-nothing allocation algorithm. However, the running time of the TransCAD system is the shortest, which is 0.143 s, and that of the Cube system is the longest, which is 0.976 s. Meanwhile, the visualization effect of the three algorithms is good, and the path allocation results can be displayed beautifully and clearly. Although the WebGIS platform runs for a long time, there is no delay. With the improvement of browser performance, the running time allocated by WebGIS will be further improved.

The results under the continuous average allocation algorithm are shown in Figure 11.  Figure 11(a) shows the running time of the system and the total flow of the road network, and Figure 11(b) shows the differences among the three systems.

Figure 11(a) shows that the path allocations of the three systems are different, and the total flow in the road network is 26493, 26843, and 26387, respectively. This is mainly because the realization means of the continuous average distribution of each system are different. Cube uses a dynamic weight number, and WebGIS uses a fixed weight coefficient. The running time of the three systems is 0.423 s, 0.872 s, and 0.241 s, respectively. WebGIS runs the shortest time. Figure 11(b) implies that there is a large error in the allocation results in the TransCAD system and Cube system because of iteration times. Accordingly, the continuous average allocation method in the proposed WebGIS has a good application traffic allocation effect and practical value.

The allocation results of the user balance algorithm are shown in Figure 12.

Figure 12 shows that the running time of the three systems is 0.157 s, 0.871 s, and 0.295 s, respectively. The average absolute errors of TransCAD and Cube systems are 23% and 5%, respectively. Besides, although the WebGIS system runs for a long time, its convergence speed is faster. The results show that the user balance allocation method in WebGIS traffic allocation is correct and has a good application effect and practical value.

### 3.4. Interaction of System Interface

In an intelligent transportation system, the system's visual display of vehicle traffic data helps dispatch vehicle traffic data. Therefore, it is necessary to display the remaining functions of the system, such as interface interaction functions. The ETC-II IoT platform is taken as the hardware terminal. Radio frequency identification identifies tag information. Zigbee controls the stepper motor to simulate electronic charging without stopping. Real-time information is transmitted through the General Packet Radio Service to verify the vehicle information query function [35, 36]. The query results are demonstrated in Table 2.

Table 2 shows that the six user information queries can display the basic vehicle information, including the specific date and time of the vehicle and the owner information. With the interactive system interface, the users can view the vehicle situation through the field monitoring terminal in real time, realizing intelligent interaction of the system.

## 4. Conclusion

In the current urban development, the increasing number of motor vehicles makes the problem of urban road congestion worsen. This article designs an urban traffic logistics management system and optimizes its interactive functions based on the basic system of WebGIS and the basic theory of road traffic assignment. The designed system can carry out road network distribution and vehicle information interactive collection, which has an important practical significance. The research results reveal that the application effect of the Dijkstra shortest path algorithm in the three path assignment algorithms is good, and the running time is 242.46 ms, 279.85 ms, and 266.86 ms, respectively. It outperforms the Floyd shortest path algorithm. The all-nothing algorithm had the shortest average total time at 264.43 ms. The running time of the remaining two algorithms is similar. Furthermore, the overall application effect of the WebGIS system is better than that of the TransCAD system and Cube system. Especially in the continuous average assignment algorithm, both the TransCAD system and Cube system have errors. The WebGIS system has no error, and the running time is only 0.241 s, which has an application value. The functional results of the interactive system show that the system can well visualize the basic information of the vehicle. The designed system has reasonable architecture, complete functions, and strong applicability. However, there are some deficiencies. The main deficiency is that the operating speed of the system cannot meet expectations. In the follow-up research, much vehicle traffic data should be collected to further optimize the model and promote the convergence speed of the system.

## Figures and Tables

**Figure 1:** B/S architecture.

**Figure 2:** Centroid and centroid connecting rod.

**Figure 3:** Main functional modules of the system.

**Figure 4:** The overall architecture of the interactive system.

**Figure 5:** Functional modules of the interactive system.

**Figure 6:** Road flow under different allocation modes.

**Figure 7:** Road impedance under different allocation modes.

**Figure 8:** Running time of the Dijkstra shortest path algorithm (a). The variation curve of the running time of different algorithms with the increase in the number of samples; (b) the variation curve of the running speed of the continuous average algorithm with the increase in the number of samples; (c) the change curve of the running speed of the user balancing algorithm with the increase in the number of samples.

**Figure 9:** Average running times under different assignment algorithms.

**Figure 10:** Path allocation under the all-and-nothing algorithm.

**Figure 11:** Path allocation under continuous average (a). The change data of the running time of the different algorithm systems and the total traffic of the road network; (b) the changing trend of the operation error rate of the different algorithm systems.

**Figure 12:** Path allocation under user balance algorithm.

**Table 1:** Basic parameters of the road network.

Design parameters	1#	2#
Distance	7534.87	7639.48
Design speed	40	40
Initial impedance	11.87	11.33
Production between two points	200	200
The attraction between the two points	200	200

**Table 2:** Summary of vehicle information.

Serial number	Date	Time	Owner's name
1	3.15	18 : 35 : 22	Z.R
2	3.15	16 : 26 : 38	Z.F.
3	3.15	20 : 18 : 53	X.T
4	3.15	18 : 15 : 43	Z.S
5	3.16	17 : 25 : 13	W.K.
6	3.16	22 : 15 : 04	Q.X. H

## Data Availability

All data are fully available without restriction.
